# To Study the Effect of Anterior Palatal Surface Modifications of Complete Denture on Speech Intelligibility Oral Perception and Cortical Brain Function Activity: An In Vivo Study

**DOI:** 10.7759/cureus.33595

**Published:** 2023-01-10

**Authors:** Prince Kumar, Challagondla Bhargavi, Shrinivas Dharaskar, Nikhat Fatima, Manjiri Salkar, Ashwini Dhopte

**Affiliations:** 1 Prosthodontics, Rama Dental College, Hospital and Research Centre, Kanpur, IND; 2 Prosthodontics, Mamata Dental College and Hospital, Khammam, IND; 3 Prosthodontics, ACPM Dental College, Dhule, IND; 4 Periodontology, Rama Dental College, Hospital and Research Centre, Kanpur, IND; 5 Prosthodontics, Mahatma Gandhi Vidyamandir’s KBH Dental College and Hospital, Nashik, IND; 6 Oral Medicine and Radiology, Rama Dental College and Research Centre, Kanpur, IND

**Keywords:** cortical brain function activity, oral perception, maxillary complete denture, anterior palatal modifications, speech

## Abstract

Background:* *The classic maxillary full denture covers the whole palate, preventing the tongue from touching the denture base tissues itself. Thus, it has deleterious effects on cortical brain function and the ability to understand spoken language.

Aim: This study aimed to determine the effect of anterior palatal surface modifications of the complete denture on speech intelligibility oral perception and cortical brain function activity.

Methods and Materials: This study compared the speech clarity, oral discernment, and cortical mind capability activity of complete denture wearers in three study groups: a) complete denture wearers with a small opening (SO) in the maxillary front palatal base; b) complete denture patients who wear regular complete denture; c) complete denture patients who did not wear complete denture; and d) complete denture patients who wear a functionally contoured modified palate (FCMP). Patients with no teeth at all underwent four phases of testing to assess their cognitive abilities and speech quality (pitch and volume). In the first phase, partial dentures were used. During phase 2, a conventional full denture was inserted. In the third phase, a palatal base denture was functionally altered. In phase 4, dentures with a little aperture at the front of the palatal base were used.

Results*:* The values of pitch and intensity of sound in category A with FCMP modification I were 180.76 ± 24.12 and 73.27 ± 9.74, respectively. On the other hand, the values of pitch and intensity of sound in category B with FCMP modification I were 185.41 ± 27.29 and 73.91 ± 8.31, respectively. The values of pitch and intensity of sound in category A with SO modification II were 188.52 ± 21.11 and 76.13 ± 5.21, respectively. On the other hand, the values of pitch and intensity of sound in category B with SO modification II were 194.59 ± 24.02 and 75.21 ± 6.12, respectively. The findings for values of pitch and intensity were statistically significant among the four phases (p < 0.001). The highest speech intelligibility and cortical brain function were observed in phase 4 in both categories A and B, with the highest scores by experts of 3.21 and 3.42, respectively.

Conclusion*: *Based on the findings of this in vivo investigation, it can be concluded that using modified dentures (modification types I and II) following denture installation improves speech intelligibility, oral perception, and cortical brain function activity.

## Introduction

Speech is considered a multi-dimensional cortical brain input that triggers linguistic associations during communication. The stomatognathic apparatus, which makes use of anatomical structures of the oral cavity as a tool, plays a significant role in speech. While the tongue, lips, and velum are considered dynamic components of speech articulation, teeth, the alveolus, and the palate are static components. These structures are essential to the production of speech sounds, and any alterations or deletions to them will have an adverse effect on those sounds [1-2]. This problem is exacerbated in edentulous individuals because the absence of all teeth and supporting structures results in poor speech sounds, poor esthetics, and difficulty chewing. Unfortunately, the most common solution for a whole mouth of missing teeth, the total denture, may have negative effects on your brain, mouth, and body [3-4].

Phonetic evaluation is typically overlooked during denture construction in favor of other important factors, including comfort, function, and esthetics. The patient's incorrect speech puts them in an uncomfortable and embarrassing scenario while wearing entire dentures. The typical belief is that patients would easily acclimatize to new dentures in a matter of weeks. However, especially for senior patients, it could take longer to adapt to alterations in the palatal outlines of maxillary full dentures. Regrettably, some patients never get used to the newer dentures and persist in having trouble articulating comprehensible sounds, particularly the sibilant sounds [5-6]. Some approaches have been proposed to increase speech intelligibility in individuals with full dentures. These include the palatographic change of the palate, the addition of roughness in the front portion of the palate, and the replication of palatal rugae in the front region. Completely covering the palate has negative effects on the oral environment, masticatory efficiency, sensorimotor function, and tongue space. Multiple types of oral sensory receptors, including proprioceptors, algethesia receptors, and thermesthesia receptors, are concentrated in the anterior palate. Speech is less audible when the tongue does not directly come in contact with the palate while speaking [7-8].

Several researchers conducted phonetics studies in connection with complete dentures to improve the clarity and understandability of speech among edentulous patients getting used to new dentures. Out of all the treatments mentioned earlier, functionally adapted palatal surface complete dentures have been shown to be the least effective in improving speech. However, there have been no notable advancements in this area. Accordingly, palatal-covering complete dentures with small openings (SOs) improved oral perception and demonstrated adequate retention force [9-10]. As the tongue makes direct contact with the palate during a speech, the cortical brain is stimulated, and clearer speech is generated. This aperture was created from the anterior maxillary incisive papilla to the third palatal folds [11]. To that end, the current study compared the actions of patients who had a complete dental replacement with a SO in the maxillary front palatal base to those who had a standard complete dental replacement, those who did not have a complete dental replacement, those who had not undergone complete dental replacement, and those who had undergone a complete dental replacement and had an FCMP.

## Materials and methods

The current in vivo investigation was conducted over a 24-month period in the department of prosthodontics with IRB number IRC/PROSTHO/2020/11. In this study, patients with total edentulousness underwent four phases of "testing to assess the quality of speech sounds (i.e., pitch and intensity) and cortical brain functioning." There was no complete denture in phase one, phase two involved a traditional complete denture, and phase three involved a functionally modified palatal base denture. In phase 4, dentures with a SO in the anterior part of the palatal base were used.

In this study, patients with total edentulousness underwent four phases of testing to assess speech intelligibility, oral perception (i.e., pitch and intensity), and cortical brain functioning. A total of 140 patients were chosen throughout the patient selection period based on inclusion and exclusion criteria. So in total 80 completely edentulous patients were included in the study proficiently. 

Inclusion criteria included a) cooperative patients; b) edentulous patients with a good level of education; c) patients with good hearing skills; d) patients who do not have any experience of silence problem or its treatment; and e) edentulous patients with a good level of education.

Exclusion criteria included a) uncooperative patients with any inherited or acquired maxillofacial deformities; b) patients with intraoral or extraoral pathologies; and c) patients with any neuromuscular disorders or visual impairments. Five participants were used in the pilot research, and from there, the sample size was established by setting the confidence interval at 10 and the confidence level at 95%.

A total of 80 people were selected as the sample size after taking into account the aforementioned factor. Two groups were created from the subjects. There were 80 people total, 40 in age group A (those 60-70) and 40 in age group B (those 70+). The institutional ethics committee gave its approval after receiving written informed consent from each patient. Each participant received a pair of upper and lower dentures manufactured to fit perfectly per Boucher's specifications. In order to lessen the horizontal forces exerted on the dentures, four acrylic teeth were reshaped and repositioned in a lingualized occlusion (LO). Noises produced by actively touching the palate with the tongue (t, d, l, and n) and sounds produced by passively touching the palate with the tongue (s, sh, ch, and JH) were used as speech stimuli in the study. Words and phrases like "Saraswati," "Tata," "Salma," "Drum," "Damru," and "Nal" are examples of the phoneme-dense speech sounds typical of the original Hindi language.

Speech samples were recorded by microphone (manufactured by Logitech Pvt. Ltd. India) with a sampling rate of 16 kHz quantized at 16 bits. All samples were recorded by an MP3 system in a soundproof room (semi-anechoic environment). For this, we turned to the Praat Sound System software. This method is a scientific tool for assessing language. Patients were instructed to sit in a soundproof room 30 cm away from the microphone. Before the actual recording started, we used a pictorial representation chart to instruct each patient.

Modifications made in a complete denture

The FCMP alteration is a type I alteration.

Oral cavity temperature

Extremely soft wax was used to create a functional shape in the palatal area of the maxillary full denture (Korecta No. 4). Patients conversed while being urged to swallow and close their mouths. Small opening (SO) modification type II at the anterior palatal base. This aperture extended from the third palatal fold to the incisive papilla. The opening was created using acrylic trimming burs, and its corners and edges were softened and beveled in the direction of the tissue. Four steps of speech analysis testing were conducted on each subject.

Assessment of the sound samples

The objective approach (quantitative analysis) and the subjective approach (qualitative analysis) were used to analyze the recorded sound recordings of each individual at various phases. The sound samples were recorded using the Praat software, which was then used for quantitative analysis. Each sample is shown using a spectrograph (sound waves). The spectrograph provided information on each recording's mean frequencies (sound pitch) and mean decibels (sound intensity/loudness). Such sound frequencies and decibel levels were tabulated and statistically analyzed to see which phase provided the clearest sound. A team of skilled speech analysts, including an ENT (ear, nose, and throat) surgeon, a speech therapist, and a prosthodontist, conducted the qualitative analysis. For each step, the intelligibility of the speech sounds produced was assessed using the five-point Likert scale. The sound recordings were played at random without any prior knowledge of the phase to prevent individual bias. The Likert scale for evaluating speech was represented by five points ranging from 0 to 4. Clear sounds were given a score of 4, normal yet slightly Puzzling sounds received a 3, requiring effort to comprehend received a 2, and indistinct sounds received a 0.

Statistical analysis

The data were collated, after which a statistical analysis was performed. The data were summarized as "mean SD" in statistical analysis (standard deviation). We can do a better job of interpreting the results of statistical analyses, and F and p values were calculated using one-way analysis of variance (ANOVA) of repeated-measures data to do between-group comparisons. The p value less than 0.05 was considered statistically significant (using a two-tailed test). Mann-Whitney test was also conducted to examine the quality of the information. Every bit of statistical work was done in SPSS (Statistical Package for the Social Sciences, IBM Version 22.0, IBM Corp., Armonk, NY).

## Results

The patients who took part in the research were classified as either Category A or Category B. Category A individuals ranged in age from 60 to 70, whereas Category B members were all 70 and over. A total of eighty patients participated in the research evenly divided between groups A and B (Table 1).

**Table 1:** Data regarding the distribution of study subjects. N, number of people

	Category A	Category B
Age group	60-70 years	≥70 years
N	40	40
Percent	50.0	50.0

The values of pitch and intensity of sound in category A without dentures were 167.31 ± 25.26 and 69.13 ± 4.12, respectively. On the other hand, the values of pitch and intensity of sound in category B without denture were 178.61 ± 24.14 and 71.24 ± 6.48, respectively. The values of pitch and intensity of sound in category A with dentures were 174.82 ± 21.46 and 68.21 ± 3.21, respectively. On the other hand, the values of pitch and intensity of sound in category B with denture were 182.24 ± 25.34 and 72.73 ± 5.79, respectively. The values of pitch and intensity of sound in category A with FCMP modification I were 180.76 ± 24.12 and 73.27 ± 9.74, respectively. On the other hand, the values of pitch and intensity of sound in category B with FCMP modification I were 185.41 ± 27.29 and 73.91 ± 8.31, respectively. The values of pitch and intensity of sound in category A with SO modification II were 188.52 ± 21.11 and 76.13 ± 5.21, respectively. On the other hand, the values of pitch and intensity of sound in category B with SO modification II were 194.59 ± 24.02 and 75.21 ± 6.12, respectively. The findings for values of pitch and intensity were statistically significant among the four phases (p < 0.001). The highest speech intelligibility and cortical brain function were observed in phase 4 in both categories A and B, with the highest scores by experts at 3.21 and 3.42, respectively (Tables 2-3).

**Table 2:** Comparison of pitch and intensity in category A and B between different phases. FCMP, functionally contoured modified palate; SO, small opening

	Pitch	Intensity
Without denture		
Category A	167.31 ± 25.26	69.13 ± 4.12
Category B	178.61 ± 24.14	71.24 ± 6.48
With denture		
Category A	174.82 ± 21.46	68.21 ± 3.21
Category B	182.24 ± 25.34	72.73 ± 5.79
FCMP modification I		
Category A	180.76 ± 24.12	73.27 ± 9.74
Category B	185.41 ± 27.29	73.91 ± 8.31
SO modification II		
Category A	188.52 ± 21.11	76.13 ± 5.21
Category B	194.59 ± 24.02	75.21 ± 6.12
Significance		
Category A	p < 0.001	p < 0.001
Category B	p < 0.001	p < 0.018

**Table 3:** Mann-Whitney U comparisons of Likert scale rating by experts for Group A and Group B. FCMP, functionally contoured modified palate; SO, small opening

Group	Category A	Category B	Mean rank of category A and category B	Significance
Without denture	1.34 ± 0.93	1.39 ± 0.72	63.49 and 60.71	p=0.865
With denture	1.97 ± 0.72	2.02 ± 0.93	60.12 and 63.09	p=0.945
FCMP modification	2.51 ± 0.81	2.44 ± 0.68	59.21 and 61.11	p=0.716
SO modification I	3.29 ± 0.87	3.41 ± 0.92	62.80 and 58.07	p=0.728

## Discussion

Several studies have been undertaken on the topic of phonetics in connection with full dentures in an effort to improve the intelligibility of speech for edentulous people adjusting to new prostheses. Functionally adapted palatal surface full dentures have been shown to be the least effective treatment for restoring a patient's ability to communicate. There haven't been any significant developments in this field, though. The palatal covering complete denture with small openings, on the other hand, was reported to improve oral perception and demonstrate appropriate retention force. Following denture wearing, the oral environment is usually altered, and the tongue has less room to move around with less efficient mastication and compromised sensorimotor function. This aperture extended from the third palatal folds to the anterior maxillary incisive papilla due to the abundance of pressure and tactile sensory sites in this area [12-15]. As a result, when the tongue directly contacts the palate while speaking, the cortical brain is stimulated, which results in clearer speech. Given this, the current study compared complete denture users with a small opening (SO) in the maxillary anterior palatal base to complete denture users without a complete denture, complete denture users without a modified palate, and complete denture users with a complete denture (FCMP).

In our study, the findings for values of pitch and intensity were statistically significant among the four phases. (p < 0.001). The highest speech intelligibility and cortical brain function were observed in phase 4 in both categories A and B, with the highest scores by experts being 3.21 and 3.42, respectively. These findings concur with those made public by Pound, Palmer, and others. Functionally changed palates were thought to be the best for producing speech sounds over time in Zakkula S et al., Kong HJ and Hansen, Tanaka H [6, 11, 14]. The patient can more readily adapt to the final denture contour by having the palatal contours of a maxillary denture tailored to the tongue. This reduces the amount of time the patient has to adjust before achieving normal enunciation [16-17]. Having no teeth or supporting structures makes this problem much worse for edentulous individuals, who often have trouble speaking clearly, have less attractive smiles, and have trouble swallowing their food. The most common dental treatment for people who have all of their teeth missing is a complete denture, however, it may have an impact on physiology, intraoral architecture, and brain activity. When making dentures, phonological evaluation is frequently neglected in favor of other crucial aspects, including comfort, functionality, and appearance [18,19]. The patient, who is wearing complete dentures, is placed in an awkward and unpleasant situation as a result of inappropriate speech. It is sometimes assumed incorrectly that patients will quickly adjust to their new dentures. People, particularly the elderly, may need more time to become used to the new palatal contours. Some individuals have difficulties speaking clearly, particularly with sibilant sounds, even after receiving new dentures [20,21].

Several techniques have been proposed in the literature to aid speech understanding in patients with full dentures. These include the insertion of roughness to the front of the palate, the reproduction of palatal rugae, and palatographic alterations. Proprioceptors, algethesia receptors, and thermesthesia receptors are only a few of the oral sensory receptors found in the front region of the palate. When the tongue does not directly contact the palate when speaking, speech is less audible [22-26]. The values of pitch and intensity of sound in this study in category A with FCMP modification I was 180.76±24.12 and 73.27±9.74 respectively. On the other hand the values of pitch and intensity of sound in category B with FCMP modification I was 185.41±27.29 and 73.91 ±8.31 respectively. The values of pitch and intensity of sound in category A with SO modification II were 188.52±21.11 and 76.13±5.21 respectively. On the other hand, the values of pitch and intensity of sound in category B with SO modification II were 194.59±24.02 and 75.21±6.12 respectively.

The functionally developed structure of the palatal contour in this study is consistent with what Tanaka found in his research [14]. These results corroborated earlier research by Zakkula S et al. Kong HJ and Hansen CA also got similar results. Research by Tanaka H, Goyal BK, and Greenstein P also produced results similar to those in our study. Studies that used a perceptive assessment of speech intelligibility, oral perception, and cortical brain functioning or spectral analysis to measure single distorted sounds reported, in accordance with the present study, that patients with a completely edentulous maxillary arch were able to speak more clearly after having dentures inserted [6,11,14,26].

The limitations of the study are the limited sample size and the fact that no other parameters affecting speech have been evaluated.

## Conclusions

Most people would agree, within the limits of this in-vivo focus, that using modified fake teeth (Change types I and II) after dental replacement improved speech clarity, oral discrimination, and cerebral mind capacity action. Full dentures with Change II (a little aperture in the front of the palatal base, or something like that) were shown to significantly improve speech clarity in comparison to Change I dentures (no opening toward the front of the dental replacement). Without any delay or adjustment time following denture placement, the natural-sounding speech was generated instantly. This design should be used to make full dentures because it has steps to reduce side strains and wear down the alveolar bone in the front of the maxilla.
